# The Shared Experience of Insured and Uninsured Patients: A Comparative Study

**DOI:** 10.1155/2022/7712938

**Published:** 2022-05-31

**Authors:** Rima Binsaeed, Mohammad Aljuaid, Shatha Alswaiti, Fatimah Alkharras, Wadi Alonazi

**Affiliations:** ^1^Management Department, College of Business Administration, King Saud University, Riyadh, Saudi Arabia; ^2^Health Administration Department, College of Business Administration, King Saud University, Riyadh, Saudi Arabia

## Abstract

**Background:**

Despite efforts to ensure equitable quality of care for all patients, a significant gap persists between the quality of care experienced by insured and uninsured patients in Saudi Arabia. This study aims to identify and compare the differences between insured and uninsured patients in terms of their experience of quality of care in a tertiary hospital.

**Methods:**

A descriptive cross-sectional study was utilized. Insured and uninsured individuals who had undergone identical medical procedures in early 2021 were identified from a public 500-bed tertiary hospital. About 350 patients participated in this study by completing an online, self-administered questionnaire, adopted by Abuosi and others in 2016, assessing six dimensions of quality of care.

**Results:**

Significant differences were reported between the quality of care experienced by insured and uninsured subjects (M = 3.37, SD = 0.525, and M = 3.06, SD = 0.452, respectively, *p*=0.001). While insured group reported high quality of care, followed by fairness of care (*r* = 0.744 and *r* = 0.675, *p* ≤ 0.001, *n* = 175), uninsured subjects experienced less fairness with low quality of care.

**Conclusions:**

The insured individuals were found to be more attentive to the quality of care offered by the hospital than their counterparts. Efforts to close the gap in quality of care should include monitoring healthcare outcomes, adopting transparency standards, and facilitating procedures to minimize barriers among patients.

## 1. Introduction

To reduce the quality chasm among society, quality of healthcare is primarily one of the cornerstone strategies implemented by health organizations worldwide [1]. Global health sector has witnessed an increasing attention to quality of health care in the last few years, especially from patients' perspectives suffering from chronic conditions. In parallel with patient-centered paradigm, health awareness toward the quality of care has also increased. Because of this heightened need for quality health care, many healthcare systems have initiated structuring their health funding by adopting universal coverage and, consequently, reducing disparities [2, 3]. Within these systems, there are normally specific groups who tend to believe that medical systems in certain social status are biased in favor of specific social segment [4]. However, such claims can only be supported by definite evaluation from the populations when they receive preferential treatment in various hospitals [5]. For the Saudi Arabian government, one of the policies put into place was to improve access equally and provide affordable services to various segments including working class and moving toward public-private partnerships [6, 7]. In terms of class, however, social inequality is also seen as a point of concern among insured and uninsured individuals when receiving quality of care within a particular health-care system [1, 8].

### 1.1. Quality of Care

According to the Institute of Medicine, the degree to which high-quality of health services are provided by increasing the level of the preferred health outcomes is collectively defined as quality of care [9]. Previous studies have confirmed that quality of care has many benefits, including ensuring patients' safety and satisfaction, preventing the overuse of health-care services, and identifying services that need to be developed [10–13]. Moreover, Michielsen and others added that those benefits include assessing quality of care facilitated in developing health insurance plans, holding individuals who fail to provide the required care accountable, and overcoming the disparities between theory and practice [14]. Assessing quality of care in health institutions is a proxy and can derive well-being through health awareness for individuals, increasing the right practices for practitioners, mainly when providing optimal services like patients' satisfaction and achieving goals, policies, and plans for organizational development [15, 16].

Health-care stakeholders have sought to identify the dimensions and factors by which quality of care is measured [17, 18]. While Fenny and colleagues claimed that these factors represent the indicators of the quality of health service, Ladhari believed that it was difficult to assess the quality of care, due to the complexity nature of healthcare and the fact that many individuals benefit from various degrees of healthcare quality [19–21]. Yarimoglu pointed out that the quality of healthcare entails providing safer, more accessible, more reliable, and more satisfactory health services to beneficiaries so that the community achieve wellness [22]. By definition, the quality of care includes the application of medical sciences and techniques to equally maximize public health benefit. Based on this, the quality is measured by balancing risks and benefits. There are core components of the quality of care that various health institutions and organizations strive to provide. One of these components is that services must be provided fairly, regardless of patients' socio-demographic characteristics such as sex, color, and insurance status. More, Steeg firmly confirmed that the provision of services should be based on how patient needs in fairly enough manner [23].

The complex nature of quality emphasizes the need to measure different experiences of quality of care in health institutions for all sorts of medical episodes. Indeed, Atinga and Baku stressed that the level of commitment to the quality of care in developing countries is low because of the existence of many socio-political restrictions that prevent the achievement of the required level of quality such as the existence of financial and human constraints [24]. Levels of variation in the quality of care are potentially attributed to resource allocation and how health insurance is financed within medical episodes [25].

### 1.2. Health Insurance

Health insurance is a method of protection against the risks of illness or injury through the provision of urgent medical care to all individuals who need it as well as compensation against temporary disability. Other studies have emphasized that health insurance is a social economic organization whose purpose is to facilitate medical service without financial impediment (cost of medical service) as a barrier between the individual and his/her access to the service [26, 27]. Consequently, health insurance is not protection against illness but security against high costs of medical service, which is sometimes called medical care insurance [28].

Globally, health insurance is proposed to be the most appropriate way to deal with the increasing cost of medical care. Abuosi emphasized that the acquisition of health insurance provides many advantages, but the degree of these advantages varies in both developed and developing economies [1]. Focusing on equity and sustainability in the European healthcare systems, Thomson and his colleagues concluded that the level of care received by uninsured individuals was low, as they received care later and at a lower level than insured individuals [29]. In Saudi Arabia (SA), Alkhamis and Miraj claimed that health-care providers pay less attention to uninsured individuals because of constraints in their financial capabilities [28].

Again, Ellis argued that increasing the volume of economic investments in healthcare, the emergence of new technologies, the development of medical technology, which is reflected in the cost of health services, and the increased cost of medicine all contribute to the increase in the cost of healthcare [30]. As such, the rise in the population is primarily related to the increased health risks of individuals, which requires the provision of healthcare for different individual ages and health conditions, resulted also in increased costs of medical care. As a result, health insurance is increasingly indicator in addressing unexpected risks and illnesses [31].

In light of the above, it can be proposed that the essence of health insurance is the achievement of the principle of social solidarity among individuals since each one should be treated according to the medical necessity. Health insurance is one of the economic pressures on both communities and individuals [26]. Previous studies have drawn a trend that health insurance relatively impacts on quality of care. Ibrahim and O'Keefe found in their study that there was no difference between the weights of infants at birth regardless of whether their parents had health insurance [32]. More, these studies also found a difference between the experiences of insured and uninsured patients regarding quality of care. The results of these previous studies have encouraged the researchers to conduct the current study to compare the experiences of the insured and uninsured patients regarding their experience of quality of care in one of the multicultural cities in SA.

### 1.3. Quality of Care and Health Insurance

Abuosi noted that there were insufficient studies regarding health insurance and quality of care and argued that previous studies that linked health insurance with the quality of care have different results. Some studies showed that health insurance leads to an improved quality of healthcare [1]. For example, Perez and others found that insured patients do receive a good level of quality of care compared to uninsured patients [33].

In addition, Nguyen and colleagues found in their Ghana-based study that although insured individuals paid for medicine and tests not included in the national health insurance scheme, they would controversially pay less compared to uninsured individuals. Other studies have proven that there is a negative impact of health insurance on the quality of care [34]. For instance, Robyn and colleagues summarized that insured patients had been waiting longer times for treatment compared to uninsured patients [35]. This result was explained by the fact that uninsured patients pay immediately to get treatment, while insured patients do not.

In contrast, others found that both insured and uninsured patients had positive experiences toward the technical quality of care, while they had negative experiences toward providers [34]. Other studies were neutral about the impact of health insurance on quality of care. For instance, health insurance had no significant impact on the quality of care for Indian patients who had a caesarean section, appendectomy, hysterectomy, or abdominal hernia surgery [36]. Methodologically, studies have focused on investigating the relationship between health insurance and quality of care by comparing the experiences of the quality of care between insured and uninsured patients, but in a certain setting not within a multicultural society [5].

### 1.4. Health Insurance in SA

In SA, government has paid special attention and priority to the healthcare sector. As a result, health services have witnessed remarkable progress over the previous ten years. The World Health Organization (WHO) has confirmed that the healthcare system in SA outperforms many other international health systems, such as Australia, and other Arab health systems, such as the UAE and Kuwait. SA's health-care system was ranked 26^th^ worldwide for a long time, but no other report was issued as there was a controversy about the methodology of the report [28]. Despite these achievements, the system faces many challenges that require policies and strategies that overcome these challenges and make concrete achievements in this area [37].

Currently, the Ministry of Health (MoH) is the main funding provider for the healthcare system in SA. Precisely, Yusuf highlighted that the most important challenge facing the MoH is the financing of health services [38]. She pointed out that expenditure on public health services laid great pressure on the government and was accompanied by a significant increase in population and employing modern technology.

Therefore, the overriding objective of this study was to compare the experiences of insured and uninsured patients in terms of the experienced quality of care while attending identical medical episodes at a tertiary hospital in SA.

## 2. Methods

This is a descriptive cross-sectional study design describing wide experiences of healthcare provided to insured and uninsured patients based on a reliable and valid self-administered questionnaire.

### 2.1. Setting and Data Collection

This study was conducted in a 500-bed facility with all medical and surgical services for insured and uninsured patients. An electronic survey (web-based) (Google docs) was emailed to particular patients admitted in the hospital and discharged within 24 hours, via patient affairs and the head nurses. The process of data collection was limited to adult patients admitted between January and May 2021. Through online survey, the questionnaire was written in Arabic and English languages. Participants completed the questionnaire, and the results ended in the principal investigator's email, but without identification of who was the subject.

### 2.2. Sampling Frame

To be legible in this study, the adults should experience identical medical episodes (whether insured or uninsured), especially in terms of procedure and treatment plan. The random-quota sample technique was conducted in specialized clinics to collect an equal number of responses, which means choosing the subject according to a specific quality. A total of 622 electronic forms were first emailed to the identified respondents by the nursing department and patient affairs.

### 2.3. Instrument and Subjects

Six dimensions of quality of care were compared among two groups (financial access, adequacy of services and resources, aspect of care, safe environment, the perceived quality of healthcare, and fairness of care). The measurement was based on 5-point Likert scale ranging from 1, very poor, to 5, very good. The instrument, adapted in this study, was developed and applied in Ghana by Abuosi and others in 2016 [1]. The questionnaire has been used by other scholars at the same studies like Chijioke in Nigeria in 2017 [21]. The instrument was examined and validated by three academic experts. Insightfully, the tool has been put through the forward back translation into the Arabic language. It was piloted and pretested on 20 participants in Arabic and English languages. To be legible for data analysis, subjects should be adults and undergo similar medical episodes, for example, patients who were treated for appendectomy were invited to participate as they were insured on uninsured. Single medical cases or nonidentical cases were excluded in this study. Each medical case for insured patient should be tallied against another medical case but for uninured patient.

### 2.4. Statistical Analysis

After data verification, they were coded, loaded, and analyzed using the SPSS program version (24.0). Descriptive statistics were used to compute means, variances, and standard deviations. Inferential tests were used like *T*-test, analysis of variance (ANOVA), Kruskal–Wallis test, and Mann–Whitney tests to measure the differences between groups. Correlation (Pearson correlation coefficient = *r*) test was used to detect the relationships between variables and determine the strength of the overall relationships between items and their dimension. The *p* value, less than 0.05, was considered as a significance level.

## 3. Results

The sociodemographic characteristics of the participants are shown in Table 1. Only 350 responses were legible for data analysis, but 50 cases were excluded because they fell under the exclusion criteria, either single medical cases or nonidentical cases. Participants were classified into two main groups, insured and uninsured patients, with 175 sample sizes for each group. The majority of the insured participants were categorized as business insurance (84.6%).

Table 1 describes the distribution of the sample according to the type of insurance and gender. Females indicated a higher number in both groups with 76% and 50.28%, respectively.

To find out the differences between insured and uninsured individuals toward dimensions of study, Table 2 is constructed based on the *t*-test. Therefore, results indicated a significant difference between insured and uninsured subjects toward all quality experience dimensions for health-care services at the hospital (*p* value less than 0.05), except in the fairness of care dimension.

To find out if there are any statistically significant differences between males and females in both insured and uninsured groups in their responses toward dimensions of study, Table 3 is constructed based on Mann–Whitney *U*-test. In both groups, there was a significant difference observed between males and females in their responses toward the adequacy of quality (*p* value less than 0.05).

To identify the correlation between quality experience dimensions, the Pearson correlation test was performed.  Table 4 shows the statistically significant relationship between all dimensions of quality experience related to the insured people.

Table 5 shows some significant relationship between all dimensions of quality experience related to the uninsured people (*p* ≤ 0.05).

## 4. Discussion

The main objective of this study was to explore equity when receiving similar medical services based on specified quality of care standards among insured and uninsured patients attending one setting. Approving a concern of the quality of care inequity, the results showed that insured individuals largely received a self-reported high to moderate levels of care than their counterparts [8, 33]. As the insured individuals were satisfied from the provided services, there was no concern mainly regarding financial access, adequacy of services and resources, technical aspects of care, safe environment, and the perceived quality of health care. This might be due to the nature of the alternative payment options available at the hospital, especially in terms of claim approval, and utilizing the technology efficiently [26].

Attracting more insured patients by implementing the quality management approaches, insured individuals were contented with services and resources offered by the hospital as it is adequate, available for integrated medical service, have a moderate level of quality, and served by qualified health-care professionals [38]. However, there are some contradictions between the results of this study and other studies. For example, the impact of the effectiveness of the health insurance system on mortality and morbidity was found neutral, indicating that both groups were treated properly and without any discrimination [39]. The results of this study are consistent with others as insured patients showed greater levels of comfort than uninsured patients [20].

In indicating that uninsured individuals received a lower level of care than insured ones, there was a dissatisfaction where uninsured persons were subjected to prolonged waiting periods, payment procedure, and a difference in treatment compared to insured patients [40–42]. On the other hand, some findings of the current study were inconsistent with other studies as the results yielded no difference in quality of care between the two groups [32, 36, 39]. The fairness of care was demonstrated similarly regardless of medical episodes as a reflection of minimum inequality among the two groups [15]. Surprisingly, findings observed that marital status, nationality, educational level, age groups, and household size did not play a key role in determining the perception of insured and insured people toward their quality experience in that hospital. Indeed, insurance coverage have an impact on overall health service utilization and consequently on personal health outcomes. During the period where the data were collected, during the COVID-19 outbreak, insured or even uninsured individuals were less likely to receive preventive medical services. Again, such variation among insured and uninsured individuals may result in unequal quality of services provided for the society [43, 44].

The study was conducted in only a tertiary hospital in Riyadh, which may limit the generalization of results. Another study in public health facilities may offer enough representation in both public and private hospitals. There is no guarantee that both groups underwent the exact procedure since the setting was not fully adopting the international classification of disease. More efforts from managers were needed to be practiced to reduce the quality chasm among individuals.

## 5. Conclusions

Moderate quality experience was demonstrated by both insured and uninsured groups; however, insured people reported higher level of experiencing quality of healthcare in a tertiary hospital than uninsured patients. The perceived quality of healthcare is pivotal in assessing quality of care for individuals. Recommendations to healthcare providers to integrate quality for both insured and uninsured can lead to improved health status and holistic welfare of society.

## Figures and Tables

**Table 1:** Distribution of the sample according to the type of insurance and gender.

		Insured (*n* = 175)		Uninsured (*n* = 175)	
		Count	%	Count	%
Type of insurance	Individual (retail)	27	15.40	0	0.00
	Business (group)	148	84.60	0	0.00

Gender	Male	42	24.00	87	49.72
	Female	133	76.00	88	50.28

**Table 2:** The experience of insured and uninsured participants towards quality of care.

Dimension	Insured (*n* = 175)		Uninsured (*n* = 175)		*p* value^*∗*^
	M.	S.	M.	S.	
Financial access	3.20	0.705	2.68	0.589	0.001
Adequacy of services and resources	3.28	0.724	2.65	0.658	001
Technical aspects of care	3.40	0.666	3.14	0.600	001
Safe environment	3.48	0.599	3.33	0.554	0.018
The perceived quality of healthcare	3.52	0.701	3.24	0.666	0.001
Fairness of care	3.24	0.617	3.12	0.555	0.055
Overall dimensions	3.37	0.525	3.06	0.4521	0.001

^*∗*^ *T*-test; M = mean; S = standard deviation.

**Table 3:** Gender difference in maintaining quality of care among the two groups.

Dimensions	Insured			Uninsured		
	M (*n* = 42)	F (*n* = 133)	*p* value	M (*n* = 87)	F (*n* = 88)	*p* value
Financial access	48.32	78.97	.006	49.08	57.91	.229
Adequacy of services and resources	53.91	78.26	.029	40.71	60.22	.008
Technical aspects of care	70.65	76.12	.622	45.50	58.90	.068
Safe environment	62.41	77.17	.186	52.10	57.07	.502
Perceived quality of healthcare	53.15	78.36	.024	50.88	57.41	.377
Fairness of care	57.00	77.86	.061	45.25	58.97	.063
Overall dimension	53.44	78.32	.026	44.06	59.29	.040

M = male; F = female.

**Table 4:** Correlation between quality experiences dimensions from insured participants' perspectives.

Insured individuals		1	2	3	4	5	6
Financial access	*r*	1					
Adequacy of services and resources	*r*	0.359^*∗∗*^	1				
	*p*	0.001					
Technical aspects of care	*r*	0.182^*∗*^	0.639^*∗∗*^	1			
	*p*	0.016	0.000				
Safe environment	*r*	0.144	0.631^*∗∗*^	0.606^*∗∗*^	1		
	*p*	0.058	0.001	0.001			
Perceived quality of healthcare	*r*	0.136	0.657^*∗∗*^	0.622^*∗∗*^	0.744^*∗∗*^	1	
	*p*	0.074	0.000	0.000	0.001		
Fairness of care	*r*	0.239^*∗∗*^	0.534^*∗∗*^	0.486^*∗∗*^	0.642^*∗∗*^	0.675^*∗∗*^	1
	*p*	0.001	0.001	0.001	0.001	0.001	

^*∗*^ = correlation is significant at the 0.05 level (2-tailed); ^*∗∗*^ = correlation is significant at the 0.01 level (2-tailed).

**Table 5:** Correlation between quality experiences dimensions from uninsured participants' perspectives.

Uninsured individuals		1	2	3	4	5	6
Financial access	*r*	1					
Adequacy of services and resources	*r*	0.413^*∗∗*^	1				
	*p*-	0.001					
Technical aspects of care	*r*	0.357^*∗*^	0.462^*∗∗*^	1			
	*p*-	0.001	0.001				
Safe environment	*r*	0.241^*∗∗*^	0.456^*∗∗*^	0.524^*∗∗*^	1		
	*p*-	0.001	0.001	0.001			
The perceived quality of healthcare	*r*	0.254^*∗∗*^	0.503^*∗∗*^	0.463^*∗∗*^	0.591^*∗∗*^	1	
	*p*-	0.001	0.001	0.001	0.001		
Fairness of care	*r*	0.270^*∗∗*^	0.469^*∗∗*^	0.411^*∗∗*^	0.393^*∗∗*^	0.617^*∗∗*^	1
	*p*-	0.001	0.001	0.001	0.001	0.001	

^*∗*^ = correlation is significant at the 0.05 level (2-tailed); ^*∗∗*^ = correlation is significant at the 0.01 level (2-tailed).

## Data Availability

The data used to support the findings of this study are available from the corresponding author upon request.

## Abbreviations

ANOVA: Analysis of variance
MoH: Ministry of Health
SA: Saudi Arabia.
